# Eating Disorders and Intrasexual Competition: Testing an Evolutionary Hypothesis among Young Women

**DOI:** 10.1100/2012/290813

**Published:** 2012-04-01

**Authors:** Riadh Abed, Sunil Mehta, Aurelio José Figueredo, Sarah Aldridge, Hannah Balson, Caroline Meyer, Robert Palmer

**Affiliations:** ^1^Ferham Clinic, Rotherham Doncaster and South Humber NHS Foundation Trust, Rotherham S61 1AJ, UK; ^2^Swallownest Court, Rotherham Doncaster and South Humber NHS Foundation Trust, Rotherham S26 4TH, UK; ^3^Department of Psychology, University of Arizona, Tucson, AZ85721, USA; ^4^Loughborough University Centre for Research into Eating Disorders, Department of Human Science, Loughborough University, Leicestershire LE11 3TU, UK; ^5^Leicester Eating Disorder Service, Leicester General Hospital, Leicester LE3 9DY, UK

## Abstract

The sexual competition hypothesis (SCH) contends that intense female intrasexual competition (ISC) is the ultimate cause of eating disorders. The SCH explains the phenomenon of the pursuit of thinness as an adaptation to ISC in the modern environment. It argues that eating disorders are pathological phenomena that arise from the mismatch between the modern environment and the inherited female adaptations for ISC. The present study has two aims. The first is to examine the relationship between disordered eating behavior (DEB) and ISC in a sample of female undergraduates. The second is to establish whether there is any relationship between disordered eating behavior and life history (LH) strategy. Participants completed a battery of questionnaires examining eating-related attitudes and behaviors, ISC, and LH strategy. A group of 206 female undergraduates were recruited. A structural equation model was constructed to analyze the data. ISC for mates was significantly associated with DEB, as predicted by the SCH. DEB was found to be predicted by fast LH strategy, which was only partially mediated by the SCH. The results of this study are supportive of the SCH and justify research on a clinical sample.

## 1. Introduction

The etiology of eating disorders is a hotly contested field of competing theories that have their origins in a diverse set of disciplines and backgrounds [1, 2]. One such discipline is evolutionary psychology which assumes that the human mind, similarly to the rest of the human organism, has been shaped by natural and sexual selection. Most existing evolutionary theories on eating disorders limit themselves to attempting to explain the causation of anorexia nervosa only (e.g., [3]) or suggest that anorexia nervosa serves an adaptive purpose, namely, reproductive suppression [4–6].

### 1.1. The Sexual Competition Hypothesis for Eating Disorders

 The SCH [7] is based on the Darwinian theory of sexual selection, the process whereby traits that lead to success in attracting high-quality mates spread preferentially within a given population. The hypothesis contends that the whole spectrum of eating disorders, as well as the pursuit of thinness, arises from intrasexual competition (ISC). ISC is an important component of sexual selection and refers to the competition amongst members of the same sex for access to members of the other sex.

 The SCH proposes that in the ancestral environment the female shape was an indicator of both reproductive history and reproductive potential and these were signaled primarily through the waist-to-hip ratio. Given the finite reproductive window for human females, who unusually amongst mammals undergo menopause, youth was a major determinant of female mate value and hence cues that display signs of youth were an important part of female ISC in the ancestral environment. Such visual cues served to attract males as well as sending powerful competitive signals to other women.

 According to the SCH, a number of factors have arisen in westernized societies that have significantly intensified female ISC [7]: declining fertility [8] leading to increasing numbers of “pseudonubile” females (preservation of the nubile appearance in older women), high levels of autonomy (i.e., ability of a given female to regulate her own reproductive behavior with minimal interference from kin), concentration of large numbers of youthful and youthful-looking women in a limited space (e.g., modern cities), relative abundance of food, and populations that are well nourished. Additionally, given the near ubiquity of good health in affluent western and westernized societies, it is contended that youth has become the primary determinant of female mate value. In such societies, the female runs the risk of increased weight and a deterioration of the nubile hourglass shape with advancing year; and as thinness has been shown to be correlated with youthfulness [9], it is contended that in western and westernized societies ISC has been carried out primarily through the display of thinness.

 A survey of over seven thousand individuals performed in ten world regions demonstrated that thin body shapes are preferred across high socioeconomic status regions [10]. Furthermore, the study found significant differences between urban and rural sites within countries and that media exposure was significantly associated with body weight ideals. In addition, it was noted that women consistently preferred thinner figures compared to men thus supporting the link between the drive for thinness and ISC.

 The SCH proposes that female ISC is the biological root for the drive for thinness, an adaptive response mechanism originally suited to the ancestral environment. The extreme version of this phenomenon manifests itself in what we call eating disorders through a process of “runaway” intrasexual competition. It is argued that the early onset eating disorder, typically anorexia nervosa with the peak age of onset being between 15 to 19 years [11], is a developmental disorder where the nubile shape is set at an abnormally low, thin level in response to the novel stimulus of the abundance of pseudonubile females in an attempt to assert their youthfulness. In contrast, bulimia nervosa that has a slightly later age of onset than anorexia nervosa [2] and rarely occurs under the age of 14 [12] is considered within SCH as the hyperactivation of the nubile program as a strategy of increasing mate value.

 Hence, SCH offers an explanation for the phenomenon of the drive for thinness, the marked female preponderance in eating disorders [13, 14], the fact that they affect primarily females of reproductive age, and it also offers an explanation for the geographical distribution of these disorders.

### 1.2. Research Supportive of the SCH

A study of 202 young American undergraduate women examined the relationship between disordered eating behavior (DEB) and ISC [15]. The study found that ISC for mates had positive direct effects on body dissatisfaction and drive for thinness and that it was the ultimate driving factor for DEB.

Further support for the SCH can be found in a study that investigated the relationship between ISC and eating restriction in university students [16]. In contrast to the male sample, exposure to competitive/high-status but not noncompetitive/low-status same-sex photos led to changes in the eating attitudes of the female sample. The study also explored the effects of intrasexual cues in homosexuals. The SCH predicts that lesbians would have a significantly lower incidence of DEB than heterosexual females as their mate attraction strategies are distinct [7]. Additionally, it is predicted that as the mate attraction strategies in homosexual men are similar to those in heterosexual females, homosexual men would have a higher incidence of DEB than heterosexual men. The study by Li et al. [16] found that heterosexual women and homosexual men, but not heterosexual men or homosexual women, reported more restrictive eating attitudes and body images concerns after exposure to competitive versus noncompetitive cues of same-sex individuals. Though not explicitly investigating clinically diagnosed eating disorders, the study found evidence consistent with the predictions of the SCH.

### 1.3. Life History (LH) Theory

In evolutionary biology, LH theory describes both species-typical and individual differences in the allocation of resources among different components of fitness, such as directing *somatic* effort towards individual survival and *reproductive* effort towards producing offspring [17]. In sexually reproducing species,* reproductive* effort is further allocated into *mating* effort, expended in mate attraction and retention, and *parental* effort, expended in promoting the survival of existing offspring [18]. *Fast* LH strategies reflect greater reproductive and mating effort and are associated in humans with impulsivity, risk-taking behavior, short-term thinking, promiscuity, lower parental investment, and little social support. *Slow* LH strategies reflect greater somatic and parental effort and are associated in humans with careful consideration of risks, long-term thinking, monogamy, extensive parental investment, and substantial social support structures.

 One theoretical implication that is relevant to DEB is that slower LH strategy should predict lower ISC. In one recent study testing the hypothesis linking DEB to LH strategy [19], a sample of female undergraduates completed a packet of questionnaires consisting of the Arizona Life History Battery, a modified version of the Eating Disorders Inventory, the behavioral regulation scales from the Behavior Rating Inventory of Executive Function, and two measures of female intrasexual competitiveness that distinguished between competition for mates and competition for status. In the path analysis reported, Executive Function was modeled as completely mediating the relation between slow life history strategy and disordered eating behavior. Surprisingly, however, the relation between female intrasexual competitiveness (competition for mates and competition for status) and disordered eating behavior was completely spurious, with executive functions serving as a common cause underlying the inhibition of both Disordered Eating Behavior and Female Intrasexual Competitiveness, which is inconsistent with certain previous findings in which they had instead been successfully modeled as causal influences [15]. The protective function of Slow Life History Strategy with respect to Disordered Eating Behavior was interpreted as residing in a higher degree of Behavioral Regulation, a type of Executive Function.

 The enhanced Behavioral Regulation, or self-control, of individuals with slow LH strategy was also protective against hazardously escalated levels of Female Intrasexual Competitiveness [19]. Therefore, we predict that if intense ISC is implicated in the drive for thinness, as the SCH predicts, then one would expect DEB to be at least *indirectly* associated with fast LH through intensified ISC amongst women. In addition to the lower levels of self-control, individuals with fast LH strategy are expected by theory to invest greater amounts of their bioenergetic resources into mating effort, which would translate directly into intrasexual competitiveness in both males and females. Whereas in males one would expect this extra mating effort to manifest itself as higher levels of aggression, both intrasexually and intersexually, including a greater inclination towards physical combat, in females one would expect this extra mating effort to take the form of more the indirect kinds of aggression typically involved in female competition [20, 21].

### 1.4. Aims

The present study intends to investigate a sample from the general female population as both the SCH and LH theory are applicable to and, therefore, testable within such a population. The study has two aims: first, to identify whether individual differences in female ISC predict DEB, and second, to determine whether individual differences in LH strategy predict female ISC, DEB, or both. As the study investigates a nonclinical population, DEB will be used as a proxy for eating disorders.

## 2. Materials and Methods

### 2.1. Participants

 Participants were 206 female students recruited via opportunity sampling at Loughborough University, UK. The women had a mean age of 20.4 years (s.d. = 1.35, range 18 to 25), and a mean body mass index (BMI) of 22.41 kg/m^2^ (s.d. = 2.72, range 15.92 to 32.03). Most participants were white (93.7%) and heterosexual (90.3%). Respondents reported being single (51.2%), in a relationship (44.9%), cohabiting, or married. Participants were not screened for current or historical eating disorders to recruit those with a full range of eating-related attitudes and behaviors [15].

### 2.2. Procedures

 Following ethical clearance (from Loughborough University Ethical Advisory Committee) and informed consent, participants completed a background information questionnaire and self-report measure of competitiveness, DEB, LH strategy, and mate values in the order presented below. Participants were offered a choice of completing either a printed version of the questionnaires or an electronic version. They were encouraged to complete the questionnaires in private and as accurately as possible and were debriefed upon completion of their questionnaires. Participants were all volunteers and did not receive incentives for participation.

### 2.3. Measures

#### 2.3.1. Measures of Female Competitiveness

 The Female Intrasexual Competitiveness Scales [15], consisted of the General Competitiveness Scale (GCS), the Female Intrasexual Competition for Mates Scale (ISC-M), and the Female Intrasexual Competition for Status Scale (ISC-S), the latter two (ISC-M and ISC-S) distinguished between intrasexual competitiveness for mates and intrasexual competitiveness for status. The GCS was incorporated in order to establish whether DEB was a manifestation of a general competitiveness rather than intrasexual competition. These two scales each contained several third-person vignettes, which consisted of questions in which participants read a situation and rated the behavior of the fictional character named Mary. Both measures contained statements requiring participants to rate their level of endorsement on 7-point Likert scales of the behavior of the hypothetical protagonist “Mary” on how likely, how appropriate, and how understandable her behavior was for each of the given scenarios. The Cronbach's alphas for each of these scales are usually about *α* = .70, which is usually considered an acceptable internal consistency reliability. Some minor adaptations were made to each of the scales with typically North American words in order to suit a UK population. A higher score on the scale indicated a higher competitiveness on that measure.

#### 2.3.2. Measures of Disordered Eating Behavior

**The Eating Disorders Inventory (EDI-S)**

EDI-S is an abbreviated version of the *EDI-2 *[22], which includes eleven subscales measuring several different aspects of disordered eating behavior: Drive for Thinness, Bulimia, Body Dissatisfaction, Ineffectiveness, Perfectionism, Interpersonal Distrust, Interoceptive Awareness, Maturity Fears, Asceticism, Impulse Regulation, and Social Insecurity. A shortened form of the *EDI-2* was used, consisting of 4 of these subscales: bulimia, body dissatisfaction, drive for thinness, and perfectionism.

**The Eating Disorders Examination Questionnaire (EDE-Q) [23]**

The *EDE-Q *is a 36-item questionnaire version of the Eating Disorders Examination interview [24]. It requires participants to either score each item from 0–6 or provide numbers for frequency items. The measure yields 4 subscale scores (Restraint, Shape Concern, Weight Concern, and Eating Concern) and a global score. High scores reflect high levels of DEB with scores greater than 4 on the subscales representing this to be at a clinical level [25]. The EDE-Q has been reported to have excellent internal consistency and 2 week test-retest reliability [26], and good concurrent validity and acceptable criterion validity in screening for DEB in community samples [25].

#### 2.3.3. Measures of Life History Strategy

**Mini-K Short Form of the ALHB (Mini-K)**

Slow LH strategy was assessed using the Mini-K Short Form [18], consisting of 20 Likert-scale items based on the 199-item Arizona Life History Battery (*ALHB)* [29], which is a battery of cognitive and behavioral indicators of life history strategy compiled and adapted from various original sources. The Mini-K correlates 0.85 with the full *ALHB* [30]. The Mini-K includes items such as, “While growing up, I had a close and warm relationship with my biological father” and “I am closely connected to and involved in my community.” The internal consistency reliability of this measure is usually about *α* = .70 in both North American and Latin-American samples.

**High-K Strategy Scale (HKSS)**

The *HKSS* is a 26-item scale based on factors documented in the literature as being indicators of a slow LH strategy [31]. It is rated by participants on a 5-point Likert scale, from “strongly disagree” to “strongly agree,” with the exception of one item. The items are internally consistent and have demonstrated acceptable reliability of about *α* = .90 in both North American and Latin American samples. The rationale for using two relatively short measures of slow LH strategy (the *Mini-K *and the *HKSS*) was to improve predictive validity compared to using one in isolation. Higher scores on these scales indicate slow LH. There is increasing support for the use of both the Mini-K and the HKSS in measuring LH strategy [32].

**Mate Value Inventory (MVI)**

The 17-item Mate Value Inventory, a measure of self-perceived possession of qualities that are considered desirable in a romantic or sexual partner, collected from the evolutionary and social psychological literature, was also included to assess how attractive individuals saw themselves, with respect to potential mates [33]. The *MVI* consists of traits empirically shown to be desirable in a romantic partner (e.g., “loyal,” “attractive face”), with five additional “distractor” items not used in the scoring. The *MVI* has demonstrated acceptable reliability of about *α* = .80 in both North American and Latin American samples. The Mate Value Inventory (MVI) is significantly correlated with the *SF-36*, which is an extensively well-validated measure of general physical and mental functioning developed by the Rand Corporation [34]. Furthermore, because producing a robust and healthy organism requires the investment of large amounts of somatic effort, as well as the receipt of large amounts of parental and nepotistic effort, we argue that high mate value also serves as an indicator of a slow LH strategy. Recent studies have indeed shown that the MVI and the Mini-K converge with other indicators upon a general LH factor [30].

### 2.4. Data Analysis

These data were subjected to a multivariate causal analysis by factor analytic structural equations modeling (*FASEM*) [35]. A *FASEM* consists of two major components: (1) a *measurement* model, and (2) a *structural* model.

 The *measurement* component of the model is essentially a confirmatory factor analysis, wherein a number of directly measured variables (called “manifest” variables or “indicators”) are related to a smaller set of hypothetical constructs (called “latent” variables or “common factors”) presumed to be underlying the correlations between them. By the exclusive prior assignment of each indicator to the theoretically specified hypothetical constructs, confirmatory factor analysis reduces the number of factor loadings needed and so enhances the efficiency of parameter estimation.

 The *structural* component of the model is essentially a path analysis between the latent constructs. Path analysis, or structural equations modeling, consists of imposing a restricted set of causal pathways, also specified *a priori*, and testing them against the correlations between constructs. A structural model that can adequately reproduce that pattern of correlations with a reduced set of hypothesized causal pathways is deemed to be superior by the principle of parsimony.

*FASEM* permits the modeling of observed correlations by any combination of theoretically specified direct effects, indirect effects, and spurious effects. In the case of the present model, the main hypotheses would be that ISC would predict DEB, and that LH strategy would predict both ISC and DEB.

## 3. Results

### 3.1. Descriptive Statistics

 The mean scores on GCS, Female ISC-M, ISC-S, and the shortened EDI are represented in Table 1.

 In Table 2, the mean scores on subscales of the EDE-Q are presented and compared to those obtained in other studies presenting normative data [27, 28]. The data from Mond et al. [27] were collected from an Australian community sample of 5255 women, ages 18–42, although only the scores for 18–22 years old are presented in Table 1. The EDE-Q subscale scores from the study by Luce et al. [28] were derived from a sample of 723 undergraduate women in the United States, ages 18–25. Using a cut-off of 4 or greater for clinical significance [27], 22% and 17.5% of the participants in the present study scored in the clinically significant range on the Shape Concern and Weight Concern subscales, respectively, slightly higher than that found in the study by Mond et al. [27] (19.4% and 11.3%) and Luce et al. [28] (14.8% and 10.2%), respectively.  Table 3 presents a comparison of the occurrence of key eating and compensatory behaviors. While objective binge episodes and excessive exercise appeared more prevalent in subjects from the present study, it should be noted that there are significant variations in the occurrence of other compensatory behaviors when comparing the results from the US and Australian samples. These variations may possibly be related to cultural and other environmental factors.

### 3.2. FASEM

Figure 1 presents the results of the *FASEM* tested on these data. The path coefficients shown are the Maximum Likelihood standardized regression weights, and all the pathways specified were statistically significant (*P* < .05). Although the chi-square value for the model was statistically significant,  *χ* ^2^(17) = 31.7840, *P* = .0160, indicating that the restricted model does not perfectly predict all the observed covariances, the practical indices of fit were considered acceptable (NFI = .922, CFI = .961). The *NFI* is the Bentler-Bonett Normed Fit Index and the CFI is the Comparative Fit Index. Indices of fit exceeding  .90 are generally considered acceptable for practical purposes [35, 36], although there is no absolute rule for these cutoffs (*cf*. [37]). Of these fit indices, however, the CFI was given greater weight in our evaluation of model adequacy because it is adjusted for model parsimony and also because it performs well with moderate-to-small sample sizes (*N* < 250), especially with Maximum Likelihood estimation [38, 39] whereas unadjusted indices, such as the NFI, may underestimate the fit of the model with smaller samples (*cf.* [37, 40]). The coefficient of determination (squared multiple correlations) for the ED-Factor was appreciable (*R* ^2^ = .221), indicating that a substantial proportion of the observed variance in reported DEB was accounted for by the specified model predictors. The standardized root mean square residual and root mean squared error of approximation were acceptably low (RMR = .0536, RMSEA = .0653), indicating a very small average absolute magnitude for the residuals, or “unexplained” components, of the observed correlations.

### 3.3. Measurement Model

 All three measures of LH converged upon a single common Slow LH factor (SLH), which loaded  .47 (*P* < .05) on the Mini-K,  .73 (*P* < .05) on the HKSS, and  .53 (*P* < .05) on the MVI-S; all three measures of competitiveness converged upon a single Competitiveness factor (COMP), which loaded  .15 (*P* < .05) on the GCS, .90 (*P* < .05) on the ISC-M, and  .47 (*P* < .05) on the ISC-S; and both measures of Disordered Eating Behavior converged upon a single outcome factor (DEB), which loaded  .67 (*P* < .05) on the EDI-S and  .93 (*P* < .05) on the EDE-Q.

### 3.4. Structural Model

 As predicted by LH theory, SLH was found to have a negative (inhibitory) effect (*β* = − .29, *P* < .05) upon COMP. COMP was found to partially mediate the effect of SLH upon DEB (*β* = −.40, *P* < .05), but a negative direct effect (*β* = −.24, *P* < .05) was also found between LH and DEB, indicating that SLH inhibits DEB by some other unmeasured mechanism as well as by the suppression of COMP.

## 4. Discussion

 This paper set out to re-examine the relationship between DEB and ISC reported by Faer et al. [15] in a sample from the general female population. The study design was extended to incorporate measures of LH strategy, thus allowing the testing of another hypothesized relationship with DEB in a sample from the general population. The results of the present study demonstrate an association between female ISC for mates and status and DEB. This is a replication of the central finding from the work of Faer et al. [15] that DEB is driven by ISC and lends support to SCH. The results also revealed a relationship between DEB and fast LH strategy. The fact that the Sexual Competition Hypothesis has now been tested in a UK population in addition to the original US population studied by Faer et al. [15] adds weight to our findings.

### 4.1. Proximate and Ultimate Causation

 The SCH is an explanation of ultimate causation for eating disorders and our findings support the contention that eating disorders measured through disordered eating behavior in a nonclinical population show a positive association with intrasexual competition. The Sexual Competition Hypothesis is essentially an environmental mismatch hypothesis that contends that the modern human urban environment of western and westernized countries exerts a pathogenic effect on certain vulnerable females and this leads some females to succumb to eating disorders in their various forms due to intense intrasexual competition.

 It may be argued that a potential weakness with SCH is that the model does not sufficiently address the question of proximate causation. Nevertheless, identifying the ultimate causation for a given disorder can be of crucial importance to the proper understanding of the nature of the disorder and could pave the way to the correct identification of previously unidentified proximate mechanisms. For example, according the present hypothesis, what we call eating disorders may in fact be disorders of female mating behavior resulting from the dysregulation of female intrasexual competition as a result of living in a modern environment that strains the evolved neurobiological systems that control mating behavior in some females beyond their level of tolerance. This implies that research on eating disorders should include the study of systems that are concerned with intrasexual competition, mate selection and mating strategies, as well as the usual issues of weight and eating control; a radical shift that would have been impossible to conceive of without considering the ultimate level of causation.

 Even before the proximate causal factors are fully understood, there is scope for the application of the current findings to clinical practice; especially if the findings from nonclinical studies are supported by those from clinical populations with eating disorders. These findings can pave the way for new methods for the assessment and treatment of eating disorders not previously considered. For example, assessments may incorporate measures of competition for mates and status as well as personal and ideal partner value. These may also be used in the design of treatment packages for eating disorders to address cognitive errors in these areas.

### 4.2. Limitations

 We acknowledge that there are some limitations due in part to the population studied. It is difficult to account for the potential bias in the self-reporting of BMI, sexual orientation, and relationship status. The study does not capture the attitudes and behaviors of other important groups, for example, males, children, and older adults in whom eating disorders may arise. The very nature of the sample meant that participants had a narrow age range. Furthermore, the subjects were undergraduates, a group generally accepted as a “healthy” population although, with regard to diagnosed eating disorders, there may be a higher incidence of pathology than the general population [41]. This may make the findings difficult to generalize to the broader general population. However, the prevalence of DEB and indeed eating disorders in higher education establishments is a focus of much research [42–44] and has led to the provision of screening and assessment facilities [45, 46]. Therefore, it could be argued that studying such a population is appropriate and worthwhile.

 Although statistically significant, the effect sizes we reported may appear weak. We believe that this is likely to be attributable to the examination of a nonclinical population in which there are relatively few “clinical cases.” We would anticipate stronger associations in clinical populations.

### 4.3. Conclusions and Future Research

 We believe we have now gathered sufficient evidence to warrant testing of the predictions of SCH on a clinical population of eating disorders sufferers. We intend to examine a clinical population with a view to determining whether there is a difference in the relationship between the particular form of eating disorder, that is, anorexia nervosa versus bulimia nervosa, and LH strategy and ISC. This was not possible in the current undergraduate sample because the different forms of DEB were not as differentiated as they would be in a clinical sample. Nevertheless, although diagnosable eating disorders that exceed the clinical cutoffs are rare, it appears that lower-level forms of disordered eating behaviors are quite common in the general population of young women and may also have an adverse, though perhaps not as severe, impact on health [19]. In addition, it would also be fruitful to explore what other mechanisms account for the residual direct effect of slow LH strategy on eating disordered behavior that is not mediated by intra-sexual competition. Future research could further explore the relationship between DEB and marital status. If DEB is related to ISC, we would anticipate different rates of DEB in single, cohabiting, and married individuals.

 Finally, if the association between ISC and LH with diagnosed eating disorders is supported by data from clinical populations, there will be scope to design future studies that test therapeutic interventions that utilize these novel insights.

## Figures and Tables

**Figure 1:** Factor Analytic Structural Equation Model for Evolutionary Psychology of Disordered Eating Behaviors in Female Undergraduates.

**Table 1:** Mean scores for the General Competitiveness Scale (GCS), Female Intrasexual Competition for Mates Scale (ISC-M), Intrasexual Competition for Status Scale (ISC-S) and shortened Eating Disorders Inventory (EDI-S).

Measure	Mean (SD)
	*n* = 206
GCS	3.42 (1.00)
ISC-M	1.92 (0.62)
ISC-S	1.88 (3.52)
EDI subscales:	
Bulimia	2.73 (3.52)
Drive for thinness	5.19 (5.42)
Perfectionism	5.55 (4.23)
Body dissatisfaction	10.25 (6.51)

SD—standard deviation.

**Table 2:** Eating Disorder Examination Questionnaire (EDE-Q) subscale scores.

	Mean (SD)		
Measure	Present study	Mond et al. [27]	Luce et al. [28]
	(18–22 age band)		
	*n* = 206	*n* = 5255	*n* = 723
EDE-Q—Restraint	1.64 (1.45)	1.29 (1.41)	1.62 (1.54)
EDE-Q—Eating Concern	1.01 (1.16)	0.87 (1.13)	1.11 (1.11)
EDE-Q—Shape Concern	2.60 (1.52)	2.29 (1.68)	2.27 (1.54)
EDE-Q—Weight Concern	2.30 (1.93)	1.89 (1.60)	1.97 (1.56)

SD—standard deviation.

**Table 3:** Proportion of women engaging in any occurrence of key eating and compensatory behaviors.

Key behavior	Any behavior (%)		
	Present study	Mond et al. [27]	Luce et al. [28]
	(18–22 age band)		
	*n* = 206	*n* = 5255	*n* = 723
Objective binge episodes	38.3	20.7	21.3
Self induced vomiting	2.9	4.8	8.8
Laxative misuse	2.4	1.3	8.3
Diuretic misuse	1.0	0.3	6.6
Excessive exercise	42.7	34.5	30.8
